The article "miR-214-3p Protects and Restores the Myocardial Tissue of Rat Myocardial Infarction Model by Targeting PTEN" was retracted in 2023. Reasons: unreliable results or conclusions; concerns about the data; concerns about the peer review; concerns about the citations.

# miR-214-3p Protects and Restores the Myocardial Tissue of Rat Myocardial Infarction Model by Targeting PTEN

**DOI:** 10.1155/2022/1175935

**Published:** 2022-07-18

**Authors:** Yuan Cheng, Qing He, Tao Jin, Na Li

**Affiliations:** ^1^Key Laboratory of Advanced Technologies of Materials, Ministry of Education, Southwest Jiaotong University, Chengdu 610031, China; ^2^Affiliated Hospital of Southwest Jiaotong University, Chengudu, China

## Abstract

Myocardial infarction (MI), which results in myocardial cell dysfunction and irreversible loss, is one of the most serious health threats today. This study was started with rats, by which the consequence of miRNA expression dysregulation to the occurrence and progression of cardiovascular diseases was explored. We first conducted miRNA sequencing on the myocardial tissues separately from myocardial infarction treatment and sham operation treatment to clarify those differently expressed miRNAs; then, our experiment of functional verification of those key miRNAs was initiated so as to dig out the molecular mechanism behind the miRNA's regulation in myocardial infarction. And it turned out that there were 32 upregulated miRNAs and 16 downregulated miRNAs according to our comparison from the myocardial infarction model group to the sham operation group; of all those upregulated, alteration in miR-214-3p expression was the most conspicuous. Overexpression of miR-214-3p greatly alleviated myocardial infarct area and ameliorated myocardial tissue structure, even reducing myocardial fibrosis and the devastation in the tissues. On the molecular level, miR-214-3p overexpression brought down both the apoptosis rate and cleaved caspase 3 expression. Besides that, we verified that PTEN is the target gene of miR-214-3p through a dual-luciferase assay. A cotransfection of miR-214-3p and PTEN brought about an obvious elevation in the myocardial infarct area, tissue damage, and fibrosis, even in the aspect of cellular apoptosis than a mere transfection of miR-214-3p. All the results above verified miR-214-3p′s effects in protecting myocardial tissues and reducing the infarct area, and it was reasonable to assume that those functions of miR-214-3p came into effect by targeting PTEN, which was then justified by the inversion to miR-214-3p′s protection via PTEN overexpression.

## 1. Introduction

According to the World Health Organization, there have been more than 6 million people worldwide suffering from myocardial infarction every year, and the mortality rate exceeds 25%. Myocardial infarction is a common coronary cardiovascular disease. At present, the mainstream treatment options include percutaneous coronary intervention, thrombolysis, and coronary artery bypass grafting. Although these therapies have improved survival after myocardial infarction to some extent, patients who do not receive these treatments have a poor prognosis.

Myocardial infarction causes cardiac cell death, resulting in damage to the heart muscle. Cardiac cells can remedy damaged tissue to some extent by regeneration, but this is not sufficient. At this time, some noncardiac cells, especially cardiac fibroblasts, would be activated, then proliferate, synthesize, and secrete collagen, forming an extracellular matrix to maintain the structural integrity and fix the damaged cardiac tissues [1]. However, excessive proliferation of myocardial fibroblasts at the sites of myocardial infarction leads to surplus accumulation of extracellular matrix, especially collagen, and increasing myocardial hardness, which is attributed to myocardial fibrosis and progressive diastolic dysfunction [2]. The purpose of this study was to explore the molecular mechanism of myocardial fibrosis development after myocardial infarction, revealing new targeted molecules for both the treatment and the diagnosis for myocardial fibrosis and providing more evidence for the correlation study of myocardial infarction.

MicroRNAs are noncoding RNAs that are only 18–25 nucleotides in length. Mature miRNAs have the ability to form RNA-induced silencing complexes with arginine proteins, which bind to the specific seed region of mRNA 3 ′-UTR, the target gene of miRNA, through base pairing, and achieve their biological function of inhibiting mRNA translation or facilitating mRNA degradation [3]. miRNAs are involved in the occurrence and the development of various diseases such as cancer, age-related cataract, and rheumatoid arthritis by affecting cell proliferation, cell differentiation, cell cycle, cell migration, and apoptosis [4]. In addition, miRNAs not only maintain normal cardiac development but are also closely related to the pathologic process of various cardiovascular diseases such as hypertension and myocardial infarction [5, 6]. Therefore, the possibility of miRNA in cardiovascular disease treatments has attracted much attention in biomedicine.

Previous studies have revealed a variety of biological functions of miR-214-3p in different cells, including the role of miR-214-3p in cardiovascular disease. Evidence from both basic and clinical studies indicates that miR-214-3p is highly expressed in hypertrophic mouse myocardium and human myocardium after myocardial infarction and in advanced heart failure, functioning as an enhancer in cell survival and antiapoptosis [7, 8]. Expression of miR-214-3p in those patients with ischemic cardiomyopathy dilated cardiomyopathy and atherosclerotic heart disease even reached 2–2.8 folds of the normal level. Evidence from in vivo experiments showed that expression of miR-214-3p in rats on the 14th day after myocardial infarction increased by 33% compared with the normal value and reached 88% on the 28th day, suggesting that miR-214-3p may affect myocardial cell proliferation, apoptosis, and ventricular remodeling after infarction by regulating its target genes.

In order to further explore the mechanism of miRNA in myocardial infarction, the differentially expressed miRNAs in the myocardial infarction rat model were detected by high-throughput sequencing in the study, and miR-214-3p was identified as a significantly differentially expressed miRNA. Furthermore, to clarify the alterations in miRNA expression during myocardial infarction and the molecular mechanism behind them, further assays on the regulatory function and the molecular mechanism of miR-214-3p were carried out on the animal level, providing a certain basis for miR-214-3p to become a new biomarker to guide the diagnosis as well as the treatment of myocardial infarction.

## 2. Methods

### 2.1. Establishment of Myocardial Ischemia Reperfusion Rat Model

Sixty male SD rats aged 6–8 weeks were provided by Chongqing Enswell Biotechnology Co., LTD. After anesthesia, the neck hair of the rats was removed, the trachea was exposed, and endotracheal intubation was performed. The breathing rate was 80 times/min, the breathing ratio was 1 : 1, and the tidal volume was 3 ml. Then the chest hair of the rat was removed, and the skin along the left margin of the sternum was cut apart; the muscles were separated, and the third and fourth intercostal muscles were opened to expose the chest. The chest wall was pulled with a hook to fully expose the heart. The left atrial appendage was removed with ophthalmic tweezers, and the left atrial appendage was gently pushed upward with cotton swabs to expose the veins between the left atrial appendage and pulmonary conus, and the secondary vein was used as a marker for ligation; a 6–0 one-time single thread was passed through the subcoronary muscle at the root of the left atrial ear 1-2 mm, with a depth of about 2 mm. Double strand line 2 was placed under the ligation line; after ligation, the color of the anterior myocardium changed from bright red to dark red rapidly and then gradually to white, indicating that the operation was successful. After 30 minutes of ischemia caused by ligation, the stitches were removed to form reperfusion, and the air in the thoracic cavity was discharged. The chest wall was sutured and stratified. After suturing, the intubation was removed and the ventilator was removed. After surgery, 80 000 units of sodium penicillin were injected intraperitoneally for 3 consecutive days to prevent infection.

### 2.2. TTC Staining

Samples were taken one week after modeling. The rat heart was manually sectioned into pieces, each 2 mm thick, immersed in 1% TTC staining solution, and bathed in water at 37°C for 30 minutes, during which the staining was improved by several times of slopping. After staining, the sections were placed in 4% paraformaldehyde fixative for 24 hours and then observed.

Measurement of the infarct areas: infarct areas (ISs) and ischemic areas (AARs) were reckoned through IPP6.0 image processing software. The percentage of infarct area was calculated according to the formula of IS/AAR%.

### 2.3. HE Staining

Samples were cleaned with PBS and fixed with 4% paraformaldehyde. In turn, these tissues were immersed in 75% ethanol, 85% ethanol, 95% ethanol, 100% ethanol I, and 100% ethanol II for 2h each. Then, the dehydrated tissues were immersed in 1/2 xylene, xylene I, and xylene II for 10 min. Transparently treated tissues were soaked with melted paraffin for 2h. The tissue in the paraffin block was cut into 2.5 *μ*m thin slices with a slicer, and the slices were laid flat on the slide. The slices were placed on a baking machine at 55°C, and the tissue slices were pressed against the slip-proof slides. The paraffin sections were immersed in xylene I, xylene II, and 1/2 xylene, respectively, for 10 min. In turn, the dewaxed paraffin sections were soaked with 100% ethanol I, 100% ethanol II, 95% ethanol I, 95% ethanol II, 85% ethanol, and 75% ethanol for 5 min each. Then the samples were rinsed 3 times with double distilled water, 2 min each time, and dyed with hematoxylin dye for 5 min. The samples were washed away with tap water for about 5 min, and then the samples were separated and decolorized with 1% alcohol hydrochloric acid to remove the excess hematoxylin staining solution in the cytoplasm. After that, the samples were dyed with eosin dye solution for 2 min and rinsed off the excess dye solution with tap water for about 1 min. Finally, the samples were washed again with distilled water, dehydrated with 95% ethanol for 2 min, then dehydrated with 100% anhydrous ethanol for 2 min; afterward, the samples were hyalinized for 5 min with xylene and then hyalinized for another 5 min with fresh xylene. The processed samples were sealed with neutral resin. Microscopic examination revealed blue nuclei and red or pink cytoplasm.

### 2.4. Masson Staining

The slices were immersed in mordant solution, kept at room temperature overnight or placed in a temperature box at 60°C for 1h for mordant, and then rinsed with water for 10 min. After that, the slices were stained with lapis lazuli blue staining drops for 3 min and washed with water twice, for 15 s each time. The samples were dyed with Mayer hematoxylin drops for 3 min and washed with distilled water twice, for 15 s each time. The sections were then differentiated with an acidic ethanol differentiation solution for several seconds until the tissues turned completely red. The differentiation was terminated with water flushing and then rinsed with distilled water for 10 min. The samples were dyed with drops of fuchsin for 10 min and washed with distilled water twice, for 15 s each time. The slices were treated with the phosphomolybdic acid solution for about 10 min, then the upper solution was dumped, and the slices were directly stained with aniline blue staining solution for 5 min without water washing. The slices were cleaned with a weak acid solution to wash away the aniline blue solution, and then the slices were covered with a weak acid working solution for 2 min. The slices were dehydrated with 95% ethanol for 30 seconds, followed by dehydration with 100% anhydrous ethanol for 2 times, the first 30 seconds and the second 1 min. Finally, the slices were hyalinized with xylene 2 times, for 2 min each time, and sealed with neutral resin. Microscopic examination showed that collagen fibers were blue, muscle fibers, cytoplasm, cellulose, keratin, and erythrocytes were red in varying degrees, and the nucleus was bluish brown.

### 2.5. TUNEL Assay on Apoptosis

The sections were washed gently with PBS, and the excess liquid around the samples was removed. A small circle with an interval of 2-3 mm from the tissue is drawn along the outer contour of the tissue with a histochemical pen for easy operation. The sample should be kept moist during the experiment, and the processed sample should be placed in a wet box to keep the sample moist. According to the 1 : 9 volume ratio, PBS was used as a diluent to dilute Proteinase K (200 *µ*g/mL) original solution, so that the final concentration was 20 *µ*g/mL. The appropriate amount of Proteinase K working solution was added to each sample to completely cover the tissues and incubated at 37°C for 20 min. The samples were washed 3 times with PBS solution, 5 min each time, and the treated samples were placed in a wet box to keep the samples moist. The excess liquid was removed from the samples, and an appropriate amount of 3% H_2_O_2_ (prepared by PBS) was dropped onto the tissues to fully infiltrate the tissues. The samples were treated at room temperature for 15 min, and then the samples were washed 3 times with PBS solution for 5 min each. The treated samples are placed in a wet box to keep them moist. The appropriate number of slides were inserted into each sample to cover the sample area and incubated with Equilibration Buffer at room temperature for 10 min. The Biotin-dUTP labeling mix and Equilibration Buffer were defrosted on ice, and the results showed that the expression of the promoter could be expressed with ct expression and Equilibration Buffer = 1 *µ*L : The 5 *µ*L: 50 *µ*L (1 : 5:50) ratio mixture is sufficient for the TdT incubation buffer for all experiments. The Equilibration Buffer was removed, and the appropriate TdT incubation buffer was added to each tissue sample and incubated at 37°C for 1 h. Sections should be kept moist and slides placed away from light. The tissue samples were immediately rinsed with PBS 4 times for 5 min each. The PBS solution around the sample was gently wiped out with a filter paper. After the slides were dried, streptavidin-HRP reaction solution (Streptavidin-HRP : TBST = 1 : 500) was added to each sample tissue and incubated at 37°C for 30 min. The sample was cleaned by PBS 3 times for 5 min each. A DAB color working solution of the appropriate amount was added to each sample, and the sections were placed under a microscope for real-time observation of color development. After a positive appearance, the slides were immediately placed in a wet box and cleaned with pure water to stop the reaction. The sections were dyed with hematoxylin solution for 1 min and washed with pure water immediately. The sections were differentiated with hematoxylin differentiation solution for about 2s and washed with pure water immediately. Then, the sections were rinsed with running water for 10 min, returned to blue, and washed with pure water. An MshotMF53 inverted microscope produced by Guangzhou Mingmei Optoelectronic Technology Co., Ltd. was used to collect images from the slices.

### 2.6. qPCR Detection on mRNA Level

After the cells were cleaned by PBS, Trizol was added, then the lysate was transferred to the new EP tube, and 200 *μ*l precooled chloroform was added per 1mL of Trizol and placed on ice for 5 min. The mixture was centrifuged at 4°C for 15 min, and the supernatant was carefully sucked out and transferred to a new EP tube. Precooled anhydrous ethanol was added to the centrifugal tube, mixed evenly, and stood. The RNA was precipitated by centrifugation at 4°C. The supernatant was discarded. Precooled 75% ethanol was added into the centrifuge tube and centrifuged at 4°C. The supernatant was completely discarded, then DEPC water was added into the dissolving centrifuge tube after standing, and mixed well; 1 *μ*L suspension was taken out for quantification and electrophoresis. Reverse transcription was performed with the Goldenstar™ RT6 cDNA Synthesis Kit Ver.2. Then use kit 2 xT5 Fast qPCR Mix (SYBR Green I) for quantitative detection. After data processing and analysis, the histogram was drawn, and the primer sequence was as follows: miR-214-3p specific reverse transcription primer: CTCAACTG GTGTCGTGGAGTCGGCAATTCAGTTGAGCCTGCCT GT; miR-214-3p-F, TCGGCAGGACAGCAGGCACAGA; miR-214-3p-R, CTCAACTGGTGTCGTGGA; PTEN-F, ACTGTAAAGCTGGGAAAG; PTEN-R, CTGAGTTGGA GGAGTAGAT; GAPDH-F, GCAAGTTCAACGGCAC AG; GAPDH-R, GCCAGTAGACTCCACGACATA.

### 2.7. Western Blot Detection on Protein Level

The frozen supernatant was taken out for protein quantification, and SDS-PAGE gels with SDS denaturation of 10% and 5% were prepared. The protein samples were mixed with the loading buffer for electrophoresis. The total protein was transferred to a polyvinylidene fluoride (PVDF) membrane by electrophoresis and incubated continuously with primary and secondary antibodies. The film was placed in a chromogenic agent, exposed, and then developed and fixed. The ImageJ software was for analyzing the gray value of the scanning results. Cleaved caspase 3 (China, AB clonal, A19654), PTEN (China, ABclonal, A19104), *β*-actin (China, ABclonal, AC026), and AS014 (China, ABclonal, AS014) were used in this study.

### 2.8. Lentivirus Packaging and Animal Model of Infection

miR-214-3p and PTEN lentiviruses were constructed and packaged by Chongqing Bio-Medicine Biotechnology Co., LTD. In animal models, 10^8^ units of the virus were injected into the tail vein immediately after modeling, once a day, and sampled after one week.

### 2.9. Dual Luciferase Assay for Target Gene Detection

The 2000bp sequence of the 3 ′UTR promoter region of PETN was synthesized and cloned into the double luciferase reporter gene vector PGL4.11-BASIC, denoted as PETN-WT-LUC2-RLUC. The binding site C1 mutation in the 2000bp sequence of the PETN promoter region was cloned into the double luciferase reporter gene vector PGL4.11-BASIC, denoted as PETN-MUT-LUC2-RLUC. 50*μ* L culture medium without antibiotics and serum was added into an EP tube with 1*μ*g (group mix) of plasmid DNA, and the mixture was gently aspirated with the pipette. Then 1.6*μ* l of nano fusion transfection reagent was added, and the transfection reagent was gently aspirated and mixed with the pipette and kept at room temperature for 5 min. Then 12 well plate cells were added. Passively buffer was added to a 12-well plate at the rate of 500*μ*L per well, and the cells were beaten with the pipette. The cells were shaken slowly on a room temperature shaker for 15 min. After that, the cell lysate was sucked into a 1.5 ml centrifuge tube, centrifuged at 12000 rpm at 4°C for 10 min, and the supernatant was transferred to a new EP tube. Then 100 *μ*L Luciferase Assay Reagent II (LARII) (Luciferase Assay Reagent Progema) working liquid was added to 96-well plates, then 20 *μ*L cell lysis solution was added, aspirated with the pipette, and the Firefly luciferase value was measured and recorded. This value is the luminescence value of the reporter gene. 100 *μ*L Stop&Glo ® Reagent (Luciferase Assay Reagent Progema) was added into the mixture and mixed with the pipette. The Renilla luciferase values were detected and recorded and deemed as the internal value.

### 2.10. Statistical Analysis

GraphPad Prism8.0 (GraphPad Software Inc, San Diego, CA, USA) was for statistical analysis and drawing, and comparison between groups was accomplished with *t*-test. #*P* < 0.05 was considered statistically significant, and ##*P* < 0.01 was considered extremely significant.

## 3. Results

### 3.1. Differentially Expressed miRNAs in the Rats with Myocardial Infarction

Firstly, this study established a rat myocardial infarction model to clarify the differential expression of miRNA in rats with myocardial infarction. TTC staining results showed that obvious infarct areas appeared in the model group (Figure 1(a)). HE staining and Masson staining results also showed that the myocardial tissue structure was significantly damaged and myocardial fibrosis was significantly increased in the model group (Figures 1(b) and 1(c)). The proportion of apoptotic cells in the model group was significantly increased by the TUNEL assay (Figure 1(d)), and cleaved caspase 3 expression was also significantly increased in the model group, which was revealed by western blot (Figure 1(e)). These results indicated that the rat myocardial infarction model has been successfully established in this study.

Subsequently, miRNA sequencing on the two groups of myocardium was to screen for differentially expressed miRNAs. The results showed that, according to our comparison of the model group with the sham group, there were 32 miRNAs upregulated and 16 miRNAs downregulated (Figure 2).

### 3.2. miR-214-3p Has the Function of Restoring Damaged Myocardial Tissues

On the basis of the results of high-throughput sequencing and further validation by qPCR detection, we found that the miR-214-3p expression in the model group was significantly lower than that in the sham group (Figure 3(a)). miR-214-3p-overexpressing and interfering lentivirus were constructed, respectively, to clarify the regulatory function of miR-214-3p (Figure 3(b)). HE staining, Masson staining, and TTC staining results showed that overexpression of miR-214-3p significantly reduces infarct sizes, improving myocardial tissue structure and alleviating myocardial fibrosis and tissue destruction (Figures 3(c) and 3(e)). Interference with miR-214-3p expression further worsens the infarct size and myocardial tissue injury. The results of TUNEL (Figure 3(f)) and western blot (Figure 3(g)) on cell apoptosis were consistent with the findings above, that is, miR-214-3p overexpression led to reduced cell apoptosis rate and decreased cleaved caspase 3 expression; however, interference to miR-214-3p further increased apoptosis rate and cleaved caspase 3 expression. In summary, miR-214-3p has the function of protecting and repairing the myocardium.

### 3.3. PTEN Is the Target Gene of miR-214-3p

In this section, we used STARBASE to predict the possible target genes of miR-214-3p. The results showed that PTEN was highly likely to be the target gene of miR-214-3p (Figure 4(a)). We detected samples from the model group and sham group and found that the expression pattern of PTEN was opposite to that of miR-214-3p (Figures 4(b) and 4(c)). In the samples with miR-214-3p overexpressed and interfered, it was found that the expression of PTEN decreased significantly after miR-214-3p was overexpressed. Interference in miR-214-3p expression significantly increased the PTEN level, but significantly decreased the expression of P13K and AKT (Figure 4(d)). Finally, the dual-luciferase assay further confirmed that PTEN was the target gene of miR-214-3p (Figure 4(e)).

### 3.4. miR-214-3p Alleviates Myocardial Infarction by PTEN

Finally, we demonstrated that miR-214-3p protects and restores myocardial infarction by targeting PTEN through the rat model of myocardial infarction co-transfected with miR-214-3p and PTEN. We found that miR-214-3p overexpression inhibited the expression of PTEN but significantly increased the P13K and AKT levels (Figure 5(a)), which effectively reduced the size of myocardial infarction and the tissue structural damage. However, the cotransfection of miR-214-3p and PTEN overexpression significantly increased the myocardial infarction areas, tissue damage, and fibrosis (Figure 5(b)); moreover, the cell apoptosis rate was also significantly higher than that of miR-214-3p overexpressed group alone (Figure 5(c)). These results suggested that miR-214-3p protects and repairs myocardium tissue by targeting PTEN inhibition, while the protective effect of miR-214-3p is withdrawn after PTEN overexpression.

## 4. Discussion

Pathologically speaking, myocardial infarction is caused by the plaques that form on the lining of the arteries, and those formed plaques cause a lack of oxygen supply, which further reduces blood flow to the heart and damages heart muscle cells [9]. Myocardial infarction causes the death of up to 1 billion cardiac cells due to ischemia. Because of the limited regenerative capacity of the adult mammalian heart, the lost cells are replaced by fibrotic tissue, which coats the cardiac structure and shapes it [10]. This shaping results in the thickening and hardening of the left ventricular wall. Many studies have confirmed myocardial fibrosis after myocardial infarction [11–13]. In this study, rats were used as experimental material to establish a myocardial infarction model by surgical ligation. After the establishment of the model, it was found that the area of myocardial infarction in mice increased, and the cardiac fibrosis and apoptosis rates increased after myocardial infarction, indicating that the rat myocardial infarction model was successfully established in this study.

A large number of studies have confirmed that the malregulation of miRNA expression is closely related to the occurrence and progression of many diseases, including cardiovascular diseases [14, 15]. In this study, the miRNA sequencing assay on the two groups of myocardial tissues was to screen for differentially expressed miRNAs to predict the differentially expressed miRNAs in our myocardial infarction models. By comparing the model group with the sham group, there were 32 miRNAs upregulated and 16 miRNAs downregulated. Among those highly downregulated miRNAs, the alteration in miR-214-3p expression was the most dramatic.

Related studies have found that miR-214-3p plays a protective role in myocardial ischemia-reperfusion injury by regulating hypoxia-inducible factor L *α* inhibitors [16]. It has been reported that HIF1AN, one of the target genes of miR-214-3p, encodes a specific asparagine hydroxylase, which leads to the hydroxylation of Asn803 in the HIF1-*α* c-terminal translation region and decreases HIF1-*α* activity by inhibiting the binding of P300 to HIF1-*α*. As soon as the expression of HIF1AN turns decreased, the activity of HIF1-*α* is increased. The miR-214-3p expression is upregulated in myocardial cells of the ischemic area, which would greatly improve cardiac systolic and restore diastolic functions, that is, reducing the damages from left ventricular systolic pressure and maximum rate of pressure rise/fall, subsequently with the damages from left ventricular end-diastolic pressure, left ventricular diameter, heart rate, and ventricular remodeling [17]. Expression of miR-214-3p in the rat myocardial cells of the ischemic area after ischemia conditioning was significantly higher than that in the myocardium directly exposed to ischemia-reperfusion injury, suggesting that ischemic conditioning could effectively upgrade the miR-214-3p protective effect on the myocardium by enhancing miR-214-3p expression. In contrast, miR-214-3p expression was significantly downregulated in those ischemic cardiomyocytes treated with ischemia-reperfusion alone, and the damages within such cardiomyocytes were relatively severe. Some scholars have found that in ischemic heart disease and heart failure, miR-214-3p expression in myocardial cells is upregulated and functions as an effective protector in myocardial ischemia-reperfusion injury. Expression of miRNA-encoded Ncx1 in the myocardial cells with miR-214-3p gene knockout is relatively upregulated when rats undergo the against-ischemia-reperfusion injury, resulting in increased calcium ion concentration in myocardial cells. In this condition, myocardial systolic protuberance is low, apoptosis is increased, and myocardial fibrosis is excessive [18]. LIU found in vivo and in vitro that upregulation of miR-214-3p induced by preconditioning could effectively improve cardiac function during ischemia-reperfusion and significantly reduce the size of myocardial infarction in experimental animals [19]. In this study, we found that the expression of miR-214-3p in the myocardial infarction model group was significantly lower than that in the sham group. Overexpression of miR-214-3p significantly reduced the size of myocardial infarction, improved the structure of myocardial tissue, and alleviated myocardial fibrosis and tissue damage. In addition, overexpression of miR-214-3p reduced the apoptosis rate as well as cleaved caspase 3 expression. This result is similar to previous studies. miRNA-488-3p has been shown to be downregulated in AMI mice and can reduce AMI-induced cardiomyocyte apoptosis by downregulating ZNF791 [20]. miR-133a and miRNA-21 have been shown to play a role in myocardial infarction diseases, such as inhibiting angiogenesis, apoptosis, fibrosis, hypertrophy, and inflammation while promoting therapeutic cardiac remodeling [21, 22].

In summary, miR-214-3p effectively protects myocardial tissue and reduces myocardial infarction, functioning as a protector and repairer for myocardium. In addition, the dual-luciferase assay in this study confirmed that PTEN was the target gene of miR-214-3p. After miR-214-3p was cotransfected with PTEN, the myocardial infarction area, tissue damage, and fibrosis notably deteriorated; besides, the apoptosis rate was evidently higher than that of the group with merely miR-214-3p overexpressed. Therefore, it can be concluded that miR-214-3p may protect and restore myocardial tissues by targeting inhibition toward PTEN, while overexpression of PTEN reverses the protective effect of miR-214-3p.

## 5. Conclusion

miR-214-3p has the functions of protecting and restoring damaged myocardium. Our experiments showed that miR-214-3p may realize the protective and restorative effects on myocardial tissues through its targeting inhibition on PTEN, while those effects of miR-214-3p would be withdrawn after the overexpression of PTEN. In this experiment, there are still areas that need to be further improved, such as the lack of in vitro experimental verification.

## Figures and Tables

**Figure 1:** Histological detection of myocardial infarction in rats. (a) TTC staining determination on the size of myocardial infarction. (b) HE staining on the myocardial tissue structure. (c) Masson's staining on myocardial fibers. (d) TUNEL staining for apoptosis estimation. (e) Western blot on cleaved caspase 3 expression.

**Figure 2:** miRNA sequencing of myocardial infarction tissues. (a) Volcano map. (b) Heat map.

**Figure 3:** Protection and restoration of miR-214-3p to myocardial tissues. (a) qPCR assay on the respective expressions of miR-214-3p in the sham group and the model group. (b) qPCR assay on the effects of overexpression and interference of miR-214-3p. (c) HE staining. (d) Masson's staining. (e) TTC staining. (f) TUNEL staining. (g) Western blot assay on cleaved caspase 3 expression.

**Figure 4:** PTEN is the target gene of miR-214-3p. (a) The STARBASE database predicted that PTEN was a possible target gene of miR-214-3p. (b) qPCR assay on the PTEN expressions in model group and sham group, respectively. (c). Western blot on the PTEN expressions in model group and sham group, respectively. (d) Western blot detection on the PTEN expressions respectively after overexpression and interference of miR-214-3p. (e) Dual luciferase detection.

**Figure 5:** miR-214-3p protects and restores damaged myocardial tissues by targeting PTEN. (a) Western blot detection on both cleaved caspase 3 and PTEN expressions separately after the overexpression of miR-214-3p and the miR-214-3p co-expression with PTEN. (b) TTC staining, HE staining, and Masson staining on the area and the tissue structures of myocardial infarction. (c) TUNEL staining.

## Data Availability

The data used to support the findings of this study are included within the article.
